# Analytical Methods for Detection of Gasotransmitter Hydrogen Sulfide Released from Live Cells

**DOI:** 10.1155/2021/5473965

**Published:** 2021-08-28

**Authors:** Fu-Shi Quan, Gi-Ja Lee

**Affiliations:** ^1^Department of Medical Zoology, College of Medicine, Kyung Hee University, Seoul 02447, Republic of Korea; ^2^Department of Biomedical Engineering, College of Medicine, Kyung Hee University, Seoul 02447, Republic of Korea

## Abstract

Hydrogen sulfide (H_2_S) plays an important role in mammals as a signaling molecule. Recently, abnormal H_2_S concentration has been associated with several pathophysiological states, such as diabetes mellitus, hypertension, Alzheimer's disease, and Parkinson's disease. As regulating H_2_S concentration can be a very prominent way of developing new drugs, many researchers have paid great attention to H_2_S research. To understand the role of H_2_S in pathophysiology and develop H_2_S-based therapies, it is necessary to measure the exact concentration of H_2_S within biological systems. But, H_2_S is volatile and can be easily oxidized. Besides, the active sites for several biological effects of H_2_S are inside the cell. Therefore, there is a need for the development of new methods for the accurate and reliable detection of H_2_S within live cells. This review provides a summary of recent developments in H_2_S detection methods for live cell analysis.

## 1. Introduction

Hydrogen sulfide (H_2_S) is a biologically relevant gaseous signaling molecule, i.e., a gasotransmitter, collectively with nitric oxide (NO) and carbon monoxide (CO) [1–3]. The endogenous production and signaling capability of H_2_S in mammalian tissues were firstly demonstrated by Abe and Kimura in 1996, showing that H_2_S is an endogenous modulator in the central nervous system [4]. Since then, there has been a dramatic shift from the belief that H_2_S works entirely as an environmental toxin to the understanding that H_2_S plays an important role in organ function and homeostasis [5]. H_2_S has been revealed to take part in the regulation of various pathophysiological conditions within mammalian systems, such as vascular tone and blood pressure [6, 7], neurotransmission [8], angiogenesis [9], cardiac function [10], various leukocytic functions [11], penile erectile function [12], and gastrointestinal tract function [13]. In general, when the concentration of H_2_S in tissues or cells is high, H_2_S is regarded as a toxic substance and its oxidation products—persulfide, sulfite, thiosulfate, and sulfate—may give rise to cytotoxic effects through inhibiting mitochondrial cytochrome C oxidase and disrupting cell energy production, resulting in tissue inflammation or DNA damage [14]. On the other hand, H_2_S at low concentrations can lead to different effects on biological processes including DNA repair and metabolism, cellular division, regulation of cell cycle, modulation of protein kinase, and organization of cytoskeletal framework [15]. But the exact physiological role of H_2_S depends on the specific circumstance, its concentration, and the interplays with other signaling molecules—NO and CO.

Recently, there have been a few trials to classify the roles of H_2_S as “H_2_S–poor” and “H_2_S-rich” under pathophysiological conditions. First, there exist a few disease states where local or systemic H_2_S deficiency either due to inhibition of H_2_S biosynthesis and/or due to increased H_2_S consumption such as asthma, diabetic vascular complications, and aging [16]. Especially, H_2_S has been known to be associated to the pathogenesis of cardiovascular diseases including hypertension [17], atherosclerosis [18], and myocardial injury [19], and the severity of these diseases is negatively related to plasma H_2_S levels [20, 21]. Besides, the mean serum H_2_S level in preeclampsia patients was significantly lower than controls [22]. And Renieris et al. suggested that H_2_S could be a potential marker for severity and final outcome of pneumonia by the SARS-CoV-2 coronavirus [23]. They showed that mortality was significantly greater among patients with a decrease of serum H_2_S levels (a cut-off point of 150.44 *μ*M) from day 1 to day 7 greater than or equal to 36%. Second, in some diseases like various forms of critical illness and multiple forms of cancer, H_2_S biosynthesis is increased due to upregulation of H_2_S-synthesizing enzymes [16]. But, there is a lack of understanding of the ideal level of H_2_S in physiology and in therapy, as well as the normal concentration range of H_2_S in circulation. One of the main obstacles is the insufficiency of an accurate and efficient detection method of H_2_S for the screening and/or identification of possible H_2_S donors and inhibitors.

H_2_S is a colorless and flammable gas with the unique odor of rotten eggs [24]. As H_2_S is a highly lipophilic molecule, it can easily penetrate the plasma membrane of all cells without any specific transporter or receptor [25]. Acute exposure to high amounts (more than 500 ppm) of H_2_S can give rise to human death [14]. H_2_S is a weak acid and easily dissolved in water with a solubility of about 80 mmol/L at 37°C [26]. Generally, it can dissociate into H^+^ and hydrosulfide anion (HS^−^), which may subsequently dissociate to H^+^ and sulfide anion (S_2_^−^) in aqueous solution. Because the two acid dissociation constants, pK_a1_ and pK_a2_, of this reaction are 6.9 and >11, respectively, H_2_S is present in the approximate ratio of 20% H_2_S and 80% HS^−^ at physiological pH [27, 28]. Nevertheless, it remains unclear whether H_2_S, HS^–^, or both are biologically active. In addition to these free H_2_S such as H_2_S gas, HS^−^, and S^2−^, H_2_S can exist in other bound sulfide pools in the biological systems including the acid-labile, alkaline-labile, and reducible sulfur, which are different from the conditions under which free H_2_S is released [29, 30]. For example, acid-labile sulfide which is derived from iron-sulfur centers in mitochondrial enzymes [27] releases H_2_S under an acidic condition (pH < 5.0). And H_2_S is released from bound sulfane sulfur under reducing conditions including excess reduced glutathionine (GSH), L-cysteine (Cys), and dithiothreitol (DTT) [27]. These complicated chemical species make it difficult to accurately measure free H_2_S in biological systems. Actually, a lot of reports do not distinguish between the three most important biologic pools of labile sulfur: free H_2_S, acid-labile, and DTT-labile sulfide, which may have completely different biological functions [31]. In addition, the volatility of H_2_S adds complications to experiments [32]. For example, there are some published reports showing that half of H_2_S can be rapidly released from culture medium in tissue culture wells within 5 min and in an even shorter time in a bubbled tissue bath [33, 34]. This may have in part contributed to large variations on the reported level of H_2_S in plasma, tissues, and certain experiments [3, 35, 36].

During the past decade, several analytical methods such as methylene blue assay [37], gas chromatography [35], and sulfide-selective electrode [7] have been developed to detect H_2_S in biological tissues or fluids. Earlier studies using the methylene blue assay reported that the H_2_S level was 26–300 *μ*M in mammalian plasma. However, later studies have shown that the high level of H_2_S may be attributed to the use of a strong acid in the methylene blue method [38, 39], because H_2_S can be released from acid-labile sulfur under a condition of a strong acid. Other methods have also been utilized to measure plasma H_2_S levels in the rat: sulfide-selective electrode showed approximately 50 *μ*M, and gas chromatography–mass spectrometry showed approximately 80 *μ*M [40]. As gas chromatography is evidently sensitive and specific, we think that it can be helpful for the detection of low physiological H_2_S levels. As a result, the large discrepancy among various reports may be attributed to the following reasons: (1) complications to experiments due to the intrinsic properties of H_2_S including the instability of sulfide, its high volatility, its great susceptibility to oxidation, and its adherence to various materials (for example, glass); (2) improper experimental conditions such as the wrong release of sulfide out of some rubbers used; (3) there were no distinction between free H_2_S, acid-labile, and DTT-labile sulfide; (4) different H_2_S levels according to age, tissue, and species; and (5) different measuring methods.

To understand biological roles of free H_2_S in health and disease state and develop H_2_S-based therapies, it is necessary to detect the exact concentration of free H_2_S within biological systems. As the active sites for various biological effects of H_2_S are inside the cell, the H_2_S level measured either in plasma or in homogenized tissue is not reflective of its cellular site of action [40]. To get more insight in their physiological roles, it is necessary to measure the H_2_S level released from cells. However, it is difficult to apply conventional methods, such as methylene blue assay, gas chromatography, and sulfide-selective electrode, to live cells owing to their destructive nature. Therefore, there had been a need for the development of novel methods for the accurate and reliable detection of endogenous free H_2_S within live cells.

Recently, a few studies regarding simple, facile, and inexpensive detection methods for the reliable detection of free H_2_S in live cells have been reported. In this review, we have focused on recent developments in H_2_S-sensing methods for live cells. We summarize the key characteristics of the analytical tools, cell types, experimental conditions for H_2_S production, and H_2_S concentration. In addition, the advantages and limitations of these methods are presented to provide a guideline for researchers to measure the H_2_S levels released from live cells.

## 2. Spectrophotometric Methods for Live Cell Analysis

Among all the reaction-based spectrophotometric methods, the methylene blue method is the traditional standard. This method was introduced by Fischer in 1883 [41] and has been utilized for H_2_S determination in many studies. As H_2_S is very volatile and can be easily oxidized, sample preparation using Zn^2+^ is generally required for the stabilization of H_2_S. In this method, the acidic condition is generally employed to liberate H_2_S from zinc sulfide complex. Subsequently, H_2_S reacts with N,N-dimethyl-p-phenylene diamine (N,N-dpd) in the presence of an oxidizing agent (usually FeCl_3_), producing methylene blue that strongly absorbs at 670 nm [42]. The absorbance is proportional to sulfide concentration. This method has been approved by the US Environmental Protection Agency as a standard method for sulfide quantization [42]. But the use of toxic and corrosive agents was the main limiting factor in terms of disturbing the application of this method to live cells.

Kartha et al. [43] reported enhanced detection of H_2_S generated in cell culture using an agar trap method (in situ methylene blue assay). As shown in Figure 1, they cultured the cells in 50 mL cell culture flasks that had a preset layer of zinc-agar on the nonadherent surface inside each flask. The H_2_S produced following incubation of the cell culture with H_2_S-releasing compounds was trapped as zinc sulfide in the zinc-agar layer. At the end of the incubation, media were carefully eliminated from the flasks without disturbing the agar layer. Then, the flasks were orientated with the agar layer, and H_2_S trapped in the agar as zinc sulfide was released and analyzed in situ utilizing a modified methylene blue reaction. This method was used to determine the activity of H_2_S-generating enzymes in intact cells, following a 24 h incubation of human endothelial-like immortalized cells Ea.hy 926 or rat vascular smooth muscle cells A10 with 1000, 3000, and 5000 *μ*M Cys. As a result, A10 cells showed about twice the activity of H_2_S-generating enzymes, compared to Ea.hy 926 cells. The authors suggested that H_2_S-generating enzymes showed different activity depending on the cell type.

The modified methylene blue-based method is inexpensive, nondestructive, adaptable to most lab settings, and more convenient than conventional methylene blue method. But the method still requires several complex steps including medium elimination, H_2_S release, and analysis of methylene blue. In addition, this method is also vulnerable to interference with colored substances, lowering its sensitivity.

Fu and Duan [44] reported a sensitive and selective method for H_2_S detection based on in situ formation of silver nanoparticles (AgNPs) on the Ag_2_S NP surface (Ag_2_S@Ag) in a layer-by-layer polyelectrolyte multilayer film using Ag amplification. The UV absorption at 430 nm showed a good linear relationship with the concentration of Na_2_S ranging from 10 nM to 5 mM. They measured free H_2_S gas generated from live liver cancer cell line HepG2 cells after treatment with Cys and pyridoxal phosphate (PLP). Although this method is sensitive and shows a wide linear range for H_2_S, it is necessary to long extra reaction time (2 h) for Ag amplification.

Ahn et al. [45] suggested a simple and cost-effective colorimetric system for selective H_2_S detection in live cells utilizing a Ag-embedded Nafion/PVP membrane applied onto a polystyrene microplate cover. The basic principle of H_2_S gas detection is the reaction between Ag and sulfide to form brown-colored Ag_2_S. A schematic illustration of the colorimetric assay is shown in Figure 2. This assay detected H_2_S release in live C6 glioma cells under stimulation of S-adenosyl methionine (SAM), thus confirming the activating effect of SAM and two substrates, Cys and homocysteine (hCys), on the pathway of cystathionine *β*-synthase- (CBS-) dependent H_2_S production [45]. Consequently, SAM-stimulated H_2_S release (10.82 ± 1.66 *μ*M) in C6 glioma cells treated with both Cys and hCys was higher compared with the H_2_S production by Cys alone (8.27 ± 0.83 *μ*M, *p* < 0.05) or without Cys and hCys (1.16 ± 0.80 *μ*M, *p* < 0.001) (Figure 2). The results were similar to the Western blot analysis of CBS expression. Using this microplate cover-based colorimetric assay, Kim et al. [46] analyzed the H_2_S-releasing properties of seven different H_2_S donors, including sodium sulfide (Na_2_S), NaHS, diallyl disulfide, diallyl trisulfide, sodium thiosulfate (Na_2_S_2_O_3_), morpholin-4-ium 4-methoxyphenyl-morpholino-phosphinodithioate (GYY4137), and Lawesson's reagent. Besides, Youness et al. [47] utilized this assay to measure the H_2_S levels released from MDA-MB-231 and MCF7 after silencing of CBS and cystathionine *γ*-lyase (CSE).

Although this method was the first report on the measurement of free H_2_S release in live cells utilizing the simple colorimetric method, the concentrations of SAM, Cys, and hCys used in this study were not physiological. But, this assay may be more helpful to explore the potential for Cys analogs and prodrugs to promote cytoprotection through the H_2_S pathway.

Zeng et al. [48] developed a colorimetric method for detection of H_2_S using gold (Au)/AgI dimeric NPs as optical probes. When Au/AgI NPs were reacted with H_2_S, AgI was changed to Ag_2_S, causing a shift in the plasmonic band of the AuNPs. The color and absorption changes were observed by naked eyes or measured by UV–vis spectroscopy (Figures 3(a) and 3(b)). In addition, the Au/AgI NPs were immobilized in agarose gels as test strips. These agarose gels were placed on the inner surface of the culture plate cover and then used for HepG2 cell culture. As a result, the H_2_S concentration was calculated as 167 nmol h^−1^ · 10^−6^ cells after treatment with Cys (2 mM) and PLP (0.5 mM) for 24 h (Figure 3(c)).

## 3. Fluorescence Detection and Imaging for Live Cell Analysis

Recently, small-molecule fluorescent probes have been attracted attention as an effective tool for detection and imaging of H_2_S in biological specimens such as tissues or cells due to their nondestructive property. The H_2_S-responsive fluorescent probes are mainly divided into four different categories depending upon their reaction types such as azide-to-amine reduction, nitro-to-amine reduction, copper sulfide precipitation, and nucleophilic addition [49, 50]. Early work in this field utilized the selective H_2_S-mediated reduction of azides and sulfonylazides, respectively, to develop first-generation reagents for fluorescence H_2_S detection [51]. Since then, Lin et al. [52] reported a family of azide-based fluorescent H_2_S indicators which had enhanced sensitivity and cellular trappability. In particular, sulfidefluor-7 acetoxymethyl ester enabled direct and real-time visualization of endogenous H_2_S release in live human umbilical vein endothelial cells under stimulation with vascular endothelial growth factor. And Yang et al. [50] developed a red-emitting fluorescent probe for H_2_S using the reduction of the azido group. This probe represented a striking fluorescence enhancement (10-fold) with a large Stokes shift (125 nm), and the detection limit was 5.7 nM. They detected exogenous and endogenous H_2_S in live HeLa cells.

Furthermore, Cheng et al. [53] developed a probe for the fluorescence switch-on detection of H_2_S, by employing dinitrophenyl ether functionality as both a fluorescence quencher and an H_2_S-reaction trigger. It was easily synthesized via nucleophilic substitution of 3,4-dinitrofluorobenzene by the BODIPY fluorophore 1. Its ability to image H_2_S in live cells was demonstrated using HeLa cells and NaHS as the H_2_S source. For specific and sensitive imaging of H_2_S in the cellular lysosome, Wu et al. [54] developed activable fluorescence nanoprobe-based quantum dots. This nanoprobe consisted of p-amino thiophenol-capped AgNPs and thioglycolic-acid-stabilized quantum dots, called QD/AgNP nanocomplexes. The detection limit of this nanoprobe was 15 nM. And they showed high ability to enter into cellular lysosome in live HeLa cells.

Compared with “turn-on” fluorescent probes, ratiometric fluorescent probes have been proposed to be more accurate for detecting H_2_S, independently of variables in quantitative analysis including variations of excitation intensity, environmental factors, light scattering, and concentration of probe [55]. An et al. [56] reported the quinoline quaternary ammonium salt derivative-based ratiometric fluorescent probe (referred to as QL-N_3_). The QL-N_3_ probe exhibited two fluorescence emission peaks at 525 and 605 nm with different excitation wavelengths of 385 and 521 nm, and the ratio between fluorescence intensities of two peaks was positively related with the H_2_S concentration. This probe could image the changes in exogenous and endogenous H_2_S in live HeLa cells.

Nevertheless, there are still several challenging issues in the development of fluorescent probes for H_2_S as follows: (i) selectivity over interfering biothiols including GSH, Cys, and hCys; (ii) high sensitivity enough to detect the endogenously produced H_2_S; (iii) fast response within a few minutes; (iv) biocompatibility including low toxicity, cell permeability, and intracellular stability; and (v) signaling in the biological optical window. Recently, Singha et al. [57] reported a two-photon fluorescent probe for H_2_S which belonged to a Michael acceptor system. They approached the selectivity issue by optimizing the electronic and steric interactions between biothiols and the probe, in addition to gaining very high sensitivity, biocompatibility, and fast response time.

Fluorescence-based detection provides excellent sensitivity, high selectivity, and real-time H_2_S monitoring not only within living cells but also within subcellular organelles. Therefore, the progress of H_2_S-specific fluorescence probes is regarded one of the fastest-growing areas in the field of H_2_S biology [58]. Although fluorescence-based detection has attracted immense attention for detecting H_2_S inside living cells, it is essential to use expensive instruments and special H_2_S probes for live cell fluorescence detection. So, it may be difficult to utilize this method in many labs.

## 4. Surface-Enhanced Raman Scattering for Live Cell Analysis

Surface-enhanced Raman spectroscopy (SERS) is a promising ultrasensitive spectral analysis technique because of its high selectivity, based on molecular fingerprinting and sensitivity, even at single-molecule detection levels [59–61]. With strong electromagnetic fields and surface chemistry enhancements, SERS can increase the original Raman signal to 10^6^ orders or more [62]. Recently, the SERS sensors have been utilized for the analysis of a variety of substances including DNA, protein, metal ions, and pesticides [63–65].

Li et al. [66] reported a novel SERS nanosensor fabricated by functionalizing AuNPs with 4-acetamidobenzenesulfonyl azide (AuNPs/4-AA) for detecting the endogenous H_2_S in live cells (Figure 4(a)). The detection was performed with SERS spectrum changes in AuNPs/4-AA coming from the reaction of H_2_S with 4-AA on AuNPs (transformation of the azide groups of 4-AA into amino groups). AuNPs/4-AA responded to H_2_S within 1 min with a 0.1 *μ*M level of sensitivity. Using SERS nanosensor, the H_2_S concentration in living glioma cells was found to have approximately 10-fold increase after 2 h stimulation of SAM, confirming that SAM can activate CBS to improve its catalytic ability to produce H_2_S. Besides, the viability of glioma cells after the addition of AuNPs/4-AA was higher than 88% at the concentration ranging from 1 to 10 nM, showing the good biocompatibility of AuNPs/4-AA (Figures 4(b) and 4(c)).

And Zhang et al. [67] proposed a smart SERS nanoprobe, Au core-4-mercaptobenzonitrile-Ag shell NP (Au@4-MBN@Ag), for detection of endogenous H_2_S in live HepG2 cells. As sulfide in the solution selectively reacted with Ag to transform Ag_2_S at room temperature, the SERS intensity of 4-MBN gradually decreased with increasing concentration of H_2_S. It showed a good linearity in the sulfide concentration ranging from 0.05 to 500 *μ*M, and a detection limit was 0.14 nM.

Though SERS has important advantages over fluorescence-based methods, such as resistance to photobleaching and phototoxicity, and narrow emission peaks for spectral multiplexing, it is still necessitated to develop H_2_S-specific SERS probes due to the difficulty in direct sensing of inorganic species. In addition, SERS require expensive instrument—Raman spectrophotometer.

## 5. Paper-Based Colorimetric Assay for Live Cell Analysis

Paper-based sensors have received great attention in the development of point-of-care (POC) diagnostics owing to the simple fabrication, cost-effectiveness, and user-friendly characteristics. The distinct properties of paper which enable passive liquid transport and compatibility with chemicals or biochemicals are the main reasons on which paper is utilized as a sensing platform [68]. In addition, the white paper is suitable for colorimetric detection because it gives strong contrast with a colored substrate [69]. So, it enables readers to check the results with the naked eye.

Rosolina et al. [70] reported a bismuth-based disposable sensor using a wet, porous, and paper-like substrate coated with alkaline bismuth hydroxide, Bi(OH)_3_. The alkaline, wet coating helped the trapping of acidic H_2_S gas and its reaction with Bi(III) species, forming colored Bi_2_S_3_ (yellow/brown). This sensor responded to ≥30 ppb H_2_S in a total volume of 1.35 L of gas. However, its alkalinity (pH 11) required special care in handling. And this sensor should be kept inside an inert gas to prevent neutralization by acidic CO_2_ in air. Carpenter et al. [71] reported a new probe using the copper(II) complex of 1-(2-pyridylazo)-2-naphthol (Cu-PAN) on the same paper-like substrate. The reaction between H_2_S gas and the copper complex led to a striking change in color from purple to yellow/orange. This color change was visible to the naked eye at the concentration as low as 30 ppb H_2_S in a 1.35 L of gas which was considered as a typical volume of human breath. They suggested that the colorimetric paper probe is easy to fabricate, cost-effective, disposable, and a green alternative to the commonly used lead acetate test papers. Recently, Ahn et al. [72] developed a rapid and simple colorimetric paper sensor using an etching-resistant effect on Ag nanoprisms. The detection principle was that Ag NPRs on the paper reacted with H_2_S gas to form Ag_2_S on their surfaces, which induced etching-resistant Ag NPRs against Cl^−^ ions. As a result, the color of Ag NPR-coated paper varied from yellow to purplish brown, depending on the concentration of H_2_S gas after KCl treatment. This H_2_S-sensing paper showed good sensitivity with a linear range of 1.03 to 32.9 *μ*M H_2_S and a fast response time of 1 min. The authors suggested that it could be utilized as a simple and reliable tool for on-site detection of H_2_S gas for quality check of dietary supplements and human breath analysis. However, the H_2_S-sensing papers mentioned above were not confirmed whether they worked properly at cell culture environment or in live cells.

Lee et al. [73] reported a new paper-based colorimetric assay by fabricating a 96-well microplate format for cell culture for sensing H_2_S gas in live cancer cells. Microplate-like hydrophobic walls designed using AutoCAD were printed using a Xerox ColorQube 8570 N printer. Wax-printed paper (Whatman grade 1 chromatography paper) consisted of 96 circular reservoirs with a 4 mm detection zone. A PVP membrane containing Ag/Nafion was coated on the H_2_S detection zones. Finally, this paper-based colorimetric assay successfully measured the difference in endogenous H_2_S level between live prostate cancer LNCaP and PC-3 cells, which showed differential expression of H_2_S-producing enzymes. Though this paper-based assay was simple, inexpensive, and feasible, it could not measure the low concentration of H_2_S released from LNCaP cells within 24 h.

## 6. Dual-Mode Detection for Live Cell Analysis

Although colorimetry-based sensing method is a simple and rapid technique for POC diagnostics and high-speed bioanalysis, the detection limit or sensitivity may be disappointing [74]. The low sensitivity can somewhat restrict the application of colorimetric methods for quantitative analysis of endogenous H_2_S in live cells under shorter time. A dual-mode detection based on colorimetry and other sensing methods such as SERS, fluorescence, or wettability can improve the sensitivity of conventional colorimetric sensors, because they give two different types of output signals covering a wider detection range [75]. Gahlaut et al. [76] introduced a dual-mode H_2_S detection combined colorimetric principle and wettability of Ag nanorod arrays on glass substrates. The surface color and water wetting properties of nanorods were found to be highly sensitive toward the H_2_S gas environment (5 ppm of gas with an exposure time of only 30 s). Together with high sensitivity and selectivity, the response time was found to be significantly low (within 5 s). The authors suggested that this method could be applied for the future study of H_2_S release from biosystems (live cells), as well as art conservation.

Zhong et al. [77] reported a colorimetric and near-infrared fluorescent probe (L) with a donor-*π*-acceptor structure derived from 4-diethylaminosalicylaldehyde and 2-(3-cyano-4,5,5-trimethylfuran-2(5H)-ylidene)malononitrile. A distinct color change of L solution from colorless to bluish-purple took place after treatment with H_2_S. Using this probe, they detected H_2_S vapor, H_2_S in water and wine samples, and H_2_S imaging in live MCF-7 cells. Besides, Paul et al. [78] reported a colorimetric and fluorescence turn-off probe 10-(4-azido phenyl)-5,5-difluoro-5h-dipyrrolo[1,2-c:1′,2′-f] [1–3] diazaborinin-4-ium-5-uide, 1, for selective detection of H_2_S. The detection limit of this probe was 0.17 *μ*M for H_2_S. They successfully detected exogenous H_2_S in live normal human oral fibroblast (NHOF) cells.

In addition, Ahn et al. [79] suggested a colorimetric and SERS-sensing system using Ag nanoplates on the paper. This dual-mode system could be helpful for detection of low concentrations of H_2_S in live cells because SERS could greatly improve the detection limit (Figure 5(a)). As a result, this simple paper assay could measure H_2_S with wider ranging from nano- to micromolar levels. And it was able to measure endogenous H_2_S in live LNCaP cells even at 8 h of incubation after cotreatment with Cys (5 mM) and hCys (1 mM) (Figure 5(b)). Besides, the viability of LNCaP cells was greater than 90% for 48 h, indicating good cell proliferation of live cells (Figure 5(c)).

Liu et al. [80] reported a ruthenium (Ru) (II) complex-based probe for colorimetric and luminescent detection and imaging of H_2_S in live cells and organisms. This Ru(II) complex was yellow color and nonluminescent in aqueous solution. But, when it reacted with H_2_S, the color of the solution changed from yellow to pink for colorimetric analysis and the emission intensity was about 65-fold increased for luminescent analysis. As this probe had low cytotoxicity and good permeability to cell membrane, it could be utilized for luminescence imaging of H_2_S in live HeLa cells.

Until now, we described the recent developments in H_2_S detection methods for live cell analysis.  Table 1 summarized some characteristics, H_2_S levels, advantages, and limitations of recently reported methods for the detection of free H_2_S from live cells. And Figures 6(a) and 6(b) show a schematic diagram of the H_2_S detection process in live cells without causing any destruction to the cells and a comparison plot of sensitivity versus accessibility of various analytical methods, respectively.

## 7. Conclusions

In this review, we have summarized the methods for the detection of H_2_S in live cells without causing any destruction to the cells. To measure H_2_S level in conventional biology, an indirect method that analyzes the expression of H_2_S synthase, such as CBS and CSE, in cell lysate or tissue homogenate using Western blot analysis is widely used. But the total analysis time for the Western blot from cell seeding is approximately 7 days including all the necessary processes such as treatment of substrates and cell lysis. To eliminate or reduce the complicated and labor-intensive analytical approach, several methods that are simple, efficient, and reliable for detection of H_2_S in live cells have been developed.

Microplate cover-based and paper-based colorimetric assays utilizing Ag/Nafion/PVP membrane can quantitatively analyze the endogenous H_2_S levels in live cancer cells, without expensive instruments and special H_2_S probes. Although these colorimetric assays are simple, easy to use, and cost-effective, they still have the limitation of low sensitivity. Recent developments in fluorescent probes for reactive sulfur species can further facilitate analysis based on fluorescence bioimaging technology. But, there are still challenging issues including high sensitivity and selectivity in the presence of many interfering biomolecules, water solubility, and low cytotoxicity. And SERS detection using H_2_S-responsive SERS probe shows great promise for the real-time monitoring of H_2_S produced in live cells, though it requires a Raman spectrophotometer. The dual-mode detection based on colorimetry and other detection methods such as SERS or fluorescence can improve the sensing performance such as high sensitivity and wide detection range, as well as easy to use. And further work for developing the highly sensitive, specific, biocompatible, and reproducible detection method is required to measure free H_2_S in live cells in the absence of additional substrates or stimulator.

## Figures and Tables

**Figure 1:** Schematic illustration of the experimental setup for H_2_S trapping method in (a) cell culture system and (b) in situ methylene blue assay. (c) Comparison of amount of H_2_S generated from Ea.hy 926 (checkered bars) and A10 (dotted bars) cells. Cells were treated with 1000, 3000, and 5000 *μ*M L-cysteine for 24 h. Reprinted from [43] with permission from publisher.

**Figure 2:** (a) Schematic illustration of microplate cover-based colorimetric assay utilizing the Ag/Nafion/PVP membrane. (b) The concentration of endogenous H_2_S production in live C6 glioma cells after treatment with s-(5′-adenosyl)-L-methionine (SAM, 2.5 mM), L-cysteine (Cys, 10 mM), and L-homocysteine (hCys, 0.5 mM) treatment in a 5% CO_2_ incubator at 37°C. Reprinted from [45] with permission from publisher.

**Figure 3:** (a) The sensing principle of Au/AgI dimeric nanoparticle-based colorimetric assay for detection of H_2_S. Photographic images of agarose gels incubated (b) with different concentrations of S^2-^ from 0 to 60 *μ*M and (c) from cell culture for 0, 8, 16, and 24 h. Reprinted from [48] with permission from publisher.

**Figure 4:** (a) Sensing mechanism of SERS nanosensors for detection of endogenous H_2_S in living cells. (b) Bright-field microscopy (A1) and dark-field microscopy (B1) images of rat C6 glioma cells after 4 h incubation with AuNPs/4-AA. (c) Cytotoxicity of different concentrations of AuNPs/4-AA in the presence and absence of NaHS after incubation of 48 h. Reprinted from [66] with permission from publisher.

**Figure 5:** (a) Schematics of the preparation of Ag nanoplate-based H_2_S-sensing paper and its principle of colorimetric and SERS dual-mode detection of H_2_S. (b) The concentration of endogenous H_2_S release from live LNCaP cells, varying with incubation times. (c) Evaluation of cellular toxicity of 5 mM L-cysteine (Cys) and 1 mM homocysteine (hCys) cotreatment in LNCaP cells. After incubation for 24 and 48 h, cellular toxicity was measured using water-soluble tetrazolium salt (WST) assay and expressed as a percentage of the control without Cys or hCys. Reprinted from [79] with permission from publisher.

**Figure 6:** (a) Schematic diagram of the H_2_S detection process in live cells. (b) Comparison plot of sensitivity versus accessibility & usability of various analytical methods for detection of H_2_S in live cells.

**Table 1:** Some characteristics and H_2_S levels of recently reported methods for the detection of free H_2_S in live cells.

Analytical methods for H_2_S		Cell types	Experimental conditions forH_2_S production	H_2_S concentration	Advantages & limitations	Ref.
Spectrophotometric method	*In situ* methylene blue assay	Rat A10 cells	24 h incubation with 1, 3, and 5 mM of Cys and 1, 2, and 5 mM NAC	40.67 ± 4.8 *μ*M (with 3 mM Cys) 51.5 ± 7.5 *μ*M (with 2 mM NAC)	(Adv.) cost-effective & adaptable to most lab. settings (Limit.) low sensitivity, several complex steps & interferences with colored substances	[43]
	Ag_2_S@AgNPs in a layer-by-layer film	HepG2 cells	2 h incubation with Cys and PLP (+Ag amplification for 2 h)	—	(Adv.) high sensitivity (10 nM) (Limit.) additional amplification time (2 h), except for the reaction time (2 h)	[44]
	Ag-embedded Nafion/PVP membrane	Rat C6 glioma cells	SAM treatment and with a combination of Cys (10 mM) and hCys (0.5 mM) for 48 h	10.82 ± 1.66 *μ*M	(Adv.) simple, facile, cost-effective, & adaptable to most lab. settings (Limit.) low sensitivity & treatment with high levels of substrates	[45]
	Au/AgI dimeric NPs	HepG2 cells	24 h incubation with 2 mM of Cys and 0.5 mM PLP	167 nmol h^−1^ · 10^−6^ cells	(Adv.) good sensitivity (500 nM) (Limit.) long response time	[48]

Fluorescence detection and imaging	Reduction of the azido group (*λ*_em_ = 610 nm)	HeLa cells	Prestimulation with 100 *μ*M of SNP (NO donor) for 60 min	—	(Adv.) high sensitivity (LOD 5.7 nM) (Limit.) only fluorescence cell imaging & long response time	[50]
	Reduction of azide to amine (*λ*_em_ = 526 nm)	HUVECs	Stimulation with VEGF (40 ng/mL) for 30 min	Intracellular fluorescence ratio ^1^*F*_f_/*F*_i_ ≈ 1.27 (vs. 1.07 of control)	(Adv.) good sensitivity (LOD 500 nM) (Limit.) long response time	[52]
	Nucleophilic cleavage of the ether bond (*λ*_em_ = 570 nm)	HeLa cells	1 h incubation with NaHS (100, 200, and 300 *μ*M)	—	(Adv.) good sensitivity (LOD 500 nM) (Limit.) only fluorescence imaging & long response time	[53]
	H_2_S-triggered disassembly of QDs/AgNP complexes (*λ*_em_ = 530 nm)	HeLa cells	Pretreatment with 300 *μ*M NaHS for 30 min	—	(Adv.) high sensitivity (LOD 15 nM) (Limit.) only fluorescence imaging & long response time	[54]
	Reduction of azide to amino group	HeLa cells	60 min incubation with Na_2_S (100 *μ*M)	The fluorescence intensity (red, 605 nm)/blue, 525 nm) ratio 2.416 (vs. 1.498 of untreated cells)	(Adv.) enhanced detection accuracy (ratiometric analysis) (Limit.) long response time	[56]

Surface-enhanced Raman scattering		Rat C6 glioma cells & human U251 MG glioma cells	SAM stimulation	Ratiometric Raman peak intensity *I*_709_/*I*_1161_: about 10-fold increase after 2 h stimulation of SAM	(Adv.) good sensitivity (LOD 0.1 *μ*M) & fast response time (1 min) (Limit.) needs specific SERS probe and expensive instrument	[66]

Paper-based colorimetric assay		LNCap cells	72 h incubation with 5 mM of Cys and 1 mM hCys	17.48 ± 3.80 *μ*M (72 h)	(Adv.) simple, low-cost, practical, & moderate sensitivity (LOD 1.4 *μ*M) (Limit.) treatment with high levels of substrates	[73]

Dual-mode detection	Colorimetry & near-IR fluorescence	MCF-7 cells	30 min incubation with NaHS (10, 50, and 100 *μ*M)	—	(Adv.) moderate sensitivity (LOD 3.09 *μ*M) & fluorescence “off-on” response (Limit.) only fluorescence imaging	[77]
	Colorimetry & fluorescence	NHOF cells	0, 20, and 60 min incubation with NaHS (10 *μ*M)	—	(Adv.) good sensitivity (LOD 0.17 *μ*M) (Limit.) only fluorescence imaging	[78]
	Colorimetry & SERS	LNCap cells	Cys (5 mM) and hCys (1 mM) treatment for 8, 16, and 24 h	0.144 ± 0.007 *μ*M (8 h) 0.211 ± 0.007 *μ*M (16 h) 2.45 ± 0.26 *μ*M (24 h)	(Adv.) high sensitivity (LOD 15 nM for SERS detection & LOD 520 nM for colorimetry) (Limit.) treatment with substrates	[79]
	Colorimetry & luminescence	HeLa cells	30 min incubation with H_2_S (200 *μ*M)	—	(Adv.) high sensitivity (LOD 53.9 nM) (Limit.) only luminescence imaging	[80]

^1^*F*_i_: initial mean fluorescence intensity; *F*_f_: final mean fluorescence intensity. Cys: L-cysteine; NAC: N-acetylcysteine; VEGF: vascular endothelial growth factor; SNP: sodium nitroprusside; HUVEC: human umbilical vein endothelial cells; SAM: s-adenosyl methionine; hCys: homocysteine. PVP: polyvinylpyrrolidone; QDs: quantum dots; AgNP: silver nanoparticle; PLP: pyridoxal phosphate; A10: vascular smooth muscle cell; NHOF: normal human oral fibroblast.
